The article "Congenital Hydronephrosis Due to Pyeloureteral Atresia: A Case Report" was retracted in 2025. Reason: concerns about the article.

# Congenital Hydronephrosis Due to Pyeloureteral Atresia: A Case Report

**DOI:** 10.7759/cureus.76664

**Published:** 2024-12-31

**Authors:** Zainab H Alowainati, Zainab H Salman, Hibah A Alhamad, Njood Alsudairy

**Affiliations:** 1 College of Medicine, Jordan University of Science and Technology, Irbid, JOR; 2 College of Medicine, Cairo University, Cairo, EGY; 3 College of Medicine, Imam Abdulrahman Bin Faisal University, Dammam, SAU; 4 Radiology, The Second Health Cluster, Jeddah, SAU

**Keywords:** abdominal ultrasound, acute intestinal obstruction, atypical presentation, fluoroscopic guidance, hydrostatic reduction, intussusception, irritability, lethargy, pediatric, target sign

## Abstract

Intussusception is a leading cause of acute intestinal obstruction in infants, typically presenting with a classic triad of intermittent abdominal pain, vomiting, and currant jelly stools. However, atypical presentations can lead to diagnostic delays, increasing the risk of complications. This report describes a seven-month-old male with an unusual presentation of lethargy and irritability, without overt gastrointestinal symptoms. Initial clinical examination, including abdominal palpation and laboratory tests, was inconclusive. However, abdominal ultrasonography revealed a subtle “target sign,” confirming intussusception despite the absence of hallmark signs. The patient underwent successful hydrostatic reduction under fluoroscopic guidance, with no pathological lead points identified. The case highlights the importance of maintaining clinical suspicion for intussusception in atypical presentations, emphasizing the critical role of early imaging in achieving timely diagnosis and favorable outcomes. Additionally, it underscores the need for vigilant post-reduction monitoring and parental education regarding recurrence.

## Introduction

Intussusception is a common cause of acute intestinal obstruction in infants and young children, characterized by the telescoping of one segment of the intestine into an adjacent segment [1]. This condition typically presents in children under two years of age and is the leading cause of intestinal obstruction in this demographic. Classic symptoms include intermittent abdominal pain, vomiting, and the passage of currant jelly stools, a sign of intestinal ischemia [1,2]. However, atypical presentations can occur and often lead to diagnostic delays, increasing the risk of complications such as bowel necrosis and perforation.

The etiology of intussusception is often idiopathic in pediatric cases, though pathologic lead points such as Meckel’s diverticulum, polyps, or lymphoid hyperplasia are occasionally identified [2,3]. Diagnosis is primarily established through imaging, with ultrasonography being the modality of choice due to its high sensitivity and specificity. The “target sign” and “pseudo-kidney sign” are hallmark findings. Early identification and treatment, typically through hydrostatic or pneumatic reduction, are critical for favorable outcomes [3,4].

This report details an infant with an atypical presentation of intussusception, highlighting the diagnostic challenges posed by non-specific symptoms such as lethargy and the absence of hallmark gastrointestinal signs. The case underscores the importance of maintaining clinical vigilance and utilizing appropriate imaging modalities in atypical presentations.

## Case presentation

This case concerns a seven-month-old male infant who presented with a 24-hour history of intermittent lethargy and reduced responsiveness, punctuated by brief periods of irritability. The parents reported that these episodes were not associated with inconsolable crying or apparent abdominal discomfort. Additionally, there were no episodes of vomiting, hematochezia, diarrhea, or significant feeding difficulties. The infant’s medical history was unremarkable, with no prior episodes of similar complaints or chronic medical conditions. His immunizations were up-to-date, and there was no recent history of gastrointestinal infections, respiratory illnesses, or dietary changes. The family history was non-contributory.

On physical examination, the infant appeared lethargic but arousable, with intermittent episodes of irritability. His vital signs were within normal limits for age, with a heart rate of 130 beats per minute, respiratory rate of 28 breaths per minute, and a temperature of 37.2°C. The abdomen was soft and non-distended, with no palpable masses or tenderness noted initially. During one of the irritability episodes, a subtle fullness was appreciated in the left lower quadrant, but no definitive sausage-shaped mass was identified. No signs of peritoneal irritation were present, and bowel sounds were hypoactive. A digital rectal examination revealed no gross blood or abnormalities, and the stool was described as normal in consistency and color.

Laboratory investigations were performed, including a complete blood count, which revealed mild leukocytosis (white blood cell count of 12,800/µL) with a neutrophilic predominance. Hemoglobin levels and platelet counts were within normal limits. C-reactive protein was mildly elevated at 10 mg/L, suggesting a possible inflammatory process. Electrolytes, renal function tests, and liver function tests were unremarkable. A urine analysis was performed to rule out a urinary tract infection, which returned normal results.

Imaging studies were initiated due to the inconclusive clinical findings and ongoing lethargy. An abdominal ultrasound revealed a “target sign” in the left lower quadrant, consistent with a structural abnormality (Figure 1). The findings were less pronounced than typically seen, and no evidence of bowel ischemia or perforation was noted. Plain abdominal radiography was obtained to rule out free air under the diaphragm, which was absent. These findings pointed towards a diagnosis of intussusception in an atypical location, despite the absence of hallmark clinical signs such as vomiting or bloody stools.

**Figure 1:** Grey-scale ultrasound image showing the classic "target sign" (arrow) of intussusception

Given the clinical and imaging findings, the differential diagnosis included intussusception, metabolic disturbances, central nervous system pathology (such as postictal states or intracranial abnormalities), and sepsis. However, the ultrasound findings conclusively identified intussusception as the primary diagnosis.

The patient was promptly referred to the pediatric surgical team for further management. After initial stabilization with intravenous fluid resuscitation and nil per os (NPO) status, a hydrostatic reduction under fluoroscopic guidance was planned. This procedure was performed successfully without complications, and post-reduction ultrasound confirmed the resolution of intussusception. No pathological lead point, such as Meckel’s diverticulum or intestinal polyp, was identified.

The patient was observed in the hospital for 24 hours following the procedure. During this period, he remained hemodynamically stable and began tolerating oral feeds without recurrence of symptoms. Serial abdominal examinations were unremarkable, and the parents were counseled extensively about the signs and symptoms of recurrence, which occurs in a small percentage of cases.

Follow-up was arranged for one week post-discharge, during which the infant was noted to have normal bowel habits and no further episodes of lethargy or irritability. A repeat ultrasound performed during the follow-up visit confirmed the absence of recurrence. The parents expressed understanding of the condition and were reassured about the favorable prognosis associated with early and effective management of intussusception.

This case highlights the importance of maintaining a high index of suspicion for intussusception in infants presenting with highly atypical symptoms, such as lethargy without overt gastrointestinal complaints. Early diagnosis and timely intervention are critical to preventing complications and ensuring a favorable outcome.

## Discussion

The presented case underscores the diagnostic challenges of intussusception when it manifests atypically, particularly in infants who do not exhibit the classic triad of abdominal pain, vomiting, and bloody stools. Atypical presentations, such as lethargy and intermittent irritability without overt gastrointestinal symptoms, can obscure clinical suspicion and delay definitive diagnosis [2-4]. This highlights the need for heightened vigilance and reliance on imaging modalities in cases where symptoms are nonspecific but concerning.

Intussusception is the most common cause of intestinal obstruction in infants, and its early identification is critical to prevent serious complications such as bowel ischemia, necrosis, or perforation. While most cases present with recognizable signs and symptoms, the absence of these hallmark features can lead to misdiagnosis or delayed diagnosis [3,5]. In this case, lethargy was the predominant symptom, a finding that is less commonly reported but can be indicative of underlying systemic compromise or hypoperfusion related to intermittent obstruction.

Ultrasound remains the gold standard for diagnosing intussusception due to its non-invasive nature, availability, and high sensitivity. The “target sign” observed in this case was instrumental in confirming the diagnosis despite the absence of classical clinical findings. In atypical cases, imaging serves as an invaluable tool for diagnosis, especially when clinical examination is inconclusive [1-3]. The early use of ultrasonography in infants with unexplained symptoms can significantly improve diagnostic accuracy and outcomes.

Management of intussusception typically involves non-surgical reduction, with hydrostatic or pneumatic methods being preferred. These approaches are effective in a majority of cases and reduce the need for invasive surgical procedures. In this case, hydrostatic reduction under fluoroscopic guidance was successfully performed, avoiding surgical intervention and its associated risks, such as infection or postoperative adhesions [2-4]. The absence of a pathological lead point, a finding consistent with idiopathic intussusception in infants, further supports the favorable prognosis observed in this patient. Idiopathic intussusception, which accounts for the majority of cases in children, is often associated with lymphoid hyperplasia, although no clear etiology was identified in this case.

Another critical aspect of care is parental education regarding the potential for recurrence, which occurs in approximately 5%-10% of cases even after successful reduction. Caregivers should be advised to monitor for any recurrence of symptoms, such as irritability, abdominal pain, or changes in bowel habits, and seek prompt medical attention [3,5]. The provision of clear discharge instructions and scheduled follow-up appointments are essential for ensuring long-term safety and addressing any subsequent concerns.

This case also contributes to the growing recognition of the varied presentations of intussusception. While the classical triad aids in diagnosis, clinicians must remain cognizant of atypical symptoms, especially in younger infants. Early imaging and timely intervention are pivotal for optimal outcomes. This report emphasizes the critical role of maintaining a broad differential diagnosis and underscores the importance of clinical vigilance, particularly when presented with nonspecific symptoms like lethargy in infants. It also highlights the need for multidisciplinary collaboration, as timely referral to pediatric surgery and the use of advanced imaging modalities were instrumental in achieving a successful outcome in this case.

## Conclusions

In conclusion, the case illustrates the complex nature of diagnosing intussusception in the absence of classic symptoms. It reinforces the value of imaging, the efficacy of non-surgical management, and the importance of post-reduction follow-up to prevent complications and ensure favorable outcomes. By presenting this atypical case, we aim to raise awareness among clinicians and support the development of more comprehensive diagnostic and management strategies for intussusception in pediatric patients.
